The article "Potent Cardioprotective Effect of the 4-Anilinoquinazoline Derivative PD153035: Involvement of Mitochondrial KATP Channel Activation" was published in 2010. Journal: PLoS One.

# Potent Cardioprotective Effect of the 4-Anilinoquinazoline Derivative PD153035: Involvement of Mitochondrial K_ATP_ Channel Activation

**DOI:** 10.1371/journal.pone.0010666

**Published:** 2010-05-17

**Authors:** Renata A. Cavalheiro, Rodrigo M. Marin, Silvana A. Rocco, Fernanda M. Cerqueira, Camille C. Caldeira da Silva, Roberto Rittner, Alicia J. Kowaltowski, Anibal E. Vercesi, Kleber G. Franchini, Roger F. Castilho

**Affiliations:** 1 Departamento de Patologia Clínica, Faculdade de Ciências Médicas, Universidade Estadual de Campinas, Campinas, Brazil; 2 Departamento de Clínica Médica, Faculdade de Ciências Médicas, Universidade Estadual de Campinas, Campinas, Brazil; 3 Departamento de Bioquímica, Instituto de Química, Universidade de São Paulo, São Paulo, Brazil; 4 Departamento de Química Orgânica, Instituto de Química, Universidade Estadual de Campinas, Campinas, Brazil; University of Illinois at Chicago, United States of America

## Abstract

**Background:**

The aim of the present study was to evaluate the protective effects of the 4-anilinoquinazoline derivative PD153035 on cardiac ischemia/reperfusion and mitochondrial function.

**Methodology/Principal Findings:**

Perfused rat hearts and cardiac HL-1 cells were used to determine cardioprotective effects of PD153035. Isolated rat heart mitochondria were studied to uncover mechanisms of cardioprotection. Nanomolar doses of PD153035 strongly protect against heart and cardiomyocyte damage induced by ischemia/reperfusion and cyanide/aglycemia. PD153035 did not alter oxidative phosphorylation, nor directly prevent Ca^2+^ induced mitochondrial membrane permeability transition. The protective effect of PD153035 on HL-1 cells was also independent of AKT phosphorylation state. Interestingly, PD153035 activated K^+^ transport in isolated mitochondria, in a manner prevented by ATP and 5-hydroxydecanoate, inhibitors of mitochondrial ATP-sensitive K^+^ channels (mitoK_ATP_). 5-Hydroxydecanoate also inhibited the cardioprotective effect of PD153035 in cardiac HL-1 cells, demonstrating that this protection is dependent on mitoK_ATP_ activation.

**Conclusions/Significance:**

We conclude that PD153035 is a potent cardioprotective compound and acts in a mechanism involving mitoK_ATP_ activation.

## Introduction

Ischemic heart disease is a global health concern, and the development of new strategies to protect the heart has attracted significant attention. Mitochondrial damage is a well known consequence of heart ischemia, and many cardioprotective drugs are targeted to this organelle [1]–[4]. Ischemia followed by reperfusion leads to increases in intracellular Ca^2+^ levels and oxidative stress, which promotes the oxidation of inner mitochondrial membrane proteins, resulting in non-selective permeabilization of this membrane. This process is known as the mitochondrial permeability transition [5], [6]. Inhibition of the permeability transition during reperfusion results in substantial prevention of structural cardiac damage and improvements of cardiac function [2]–[4], [7]–[9].

In addition to undergoing damage during ischemia, mitochondria have been uncovered as important sites for signaling processes related to ischemia and myocardial protection. Ischemic preconditioning, a protocol in which short periods of ischemia protect against subsequent longer damaging ischemic periods [10], involves changes in mitochondrial reactive oxygen species release and ion transport [11]–[14]. More specifically, activation of ATP-sensitive K^+^ channels in mitochondria (mitoK_ATP_) is a necessary step for cardioprotection promoted by ischemic preconditioning [15], [16]. MitoK_ATP_ activation is also necessary for cardioprotection promoted by adenosine, respiratory chain inhibitors and some anesthetics [2], [12], [17]–[19]. Activation of phosphoinositide 3 kinase (PI3K)-AKT has been implicated as an upstream event in the mitoK_ATP_ activation in preconditioning [20], [21].

Epidermal growth factor (EGF) tyrosine kinase 2 is an important survival factor for human cardiomyocytes [22], and EGF receptor tyrosine kinase activity has been also implicated in the pathogenesis of cardiovascular disorders [23]–[27]. Here, we tested the possible cardioprotective effects of PD153035, a 4-anilinoquinazoline derivative developed as an EGF receptor tyrosine kinase inhibitor [28]. We found that PD153035 is a potent cardioprotective agent in perfused rat hearts and cardiac HL-1 cells. Interestingly, we demonstrate that cardioprotection by PD153035 is associated with mitoK_ATP_ activation, and provide evidence that this drug may be a direct agonist of this channel.

## Materials and Methods

### Materials and laboratory animals

All reagents used were of analytical grade or better, and deionized water was used for all aqueous solutions. PD153035 [4-*N*-(3′-bromophenylamino)-6,7-dimethoxyquinazoline hydrochloride] (>99% purity) was synthesized as previously described [29]. PD153035 solutions were prepared daily, in DMSO.

Male Wistar rats were obtained from the UNICAMP Central Animal Breeding Facilities (Campinas, Brazil). Protocols used were approved by the local Committee for Ethics in Animal Research, and conformed with the Guide for the Care and Use of Laboratory Animals published by the US National Institutes of Health (NIH Publication No. 85-23, revised 1996).

### Isolated heart preparations

Male Wistar rats weighing 200–250 g were anesthetized with pentobarbital sodium (50 mg/kg i.p.) and placed on a temperature-controlled surgical table. After injection of heparin sodium (500 U/kg i.v.), hearts were removed [30], and the aorta was cannulated with a 20-gauge catheter positioned ∼2 mm above the coronary ostia. Hearts were perfused with HEPES buffer (137 mM NaCl, 5 mM KCl, 1.2 mM MgCl_2_, 1.5 mM CaCl_2_, 6 mM glucose, 2 U/L insulin, 0.0001% xylocaine, 1000 U/L heparin and 20 mM HEPES, pH 7.4) bubbled with 100% O_2_ at a constant pressure of 70 mmHg, at 37°C. Where indicated, PD153035 was added to the perfusion buffer and present during the full perfusion protocol, from the stabilizing period until the end of the reperfusion. Control hearts were perfused with the same quantity as perfused hearts of DMSO, which remained under 0.01%. Left ventricular diastolic pressure was kept constant at 5 mmHg and continuously monitored (WinDaq Software, DATAQ Instruments, Inc., Akron, OH, USA) through a water-filled latex balloon inserted into the lumen of the left ventricle via the left atrium. The distal end of the balloon-attached catheter was connected to a pressure transducer for intraventricular pressure monitoring. Ventricular function was determined from left ventricular pressure measurements.

### Cell cultures

Murine atrial HL-1 cells were developed and kindly donated by Prof. William C. Claycomb (Louisiana State University, New Orleans, LO, USA). These cells maintain their cardiac phenotype during extended passages, present ordered myofribrils, cardiac-specific junctions and several voltage-dependent currents that are characteristic of a cardiac myocyte phenotype [31]. Furthermore, HL-1 cells present conserved preconditioning mechanisms dependent on protein kinase C and K^+^ channel activation [32] and ischemic damage dependent on the mitochondrial permeability transition [8]. For routine growth, HL-1 cells were maintained in T-75 flasks at 37°C in an atmosphere of 5% CO_2_ in Claycomb medium (JRH Biosciences, Lenexa, KS, USA) supplemented with 0.1 mM norepinephrine, 100 U/mL and 100 µg/mL penicillin/streptomycin, 2 mM glutamine and 10% fetal bovine serum. Experiments were conducted when the cultures reached 100% confluence, after trypsinization and resuspension of the cells in a standard buffer (pH = 7.4) containing (in mmol/L): NaCl, 137; Hepes, 5; glucose, 22; taurine, 20; creatine, 5; KCl, 5.4; MgCl_2_, 1; sodium pyruvate, 5 and CaCl_2_, 1 [8], [14]. Cells were maintained in suspension during the experimental protocols, at a concentration ∼1.5×10^6^ cells/mL.

### Simulated ischemia/reperfusion (cyanide/aglycemia) in cultured HL-1 cells

Ischemia was simulated by metabolic inhibition and substrate deprivation using 10 mM potassium cyanide and 2 mM 2-deoxyglucose, added to standard buffer devoid of glucose and pyruvate. The joint presence of cyanide and deoxyglucose inhibits oxygen consumption in these cells by at least 95% (H.T. Facundo and A.J. Kowaltowski, unpublished observations), in a reversible manner. HL-1 myocytes were incubated under cyanide/aglycemia during 60 min followed by 5 min centrifugation and re-suspension of the cell pellet in control buffer for simulated reperfusion. Where indicated, 10 nM PD153035, 0.05% DMSO (controls) and/or 60 µM 5HD were present during the 20 min pre-incubation period before cyanide/aglycemia. Control HL-1 myocytes were incubated with standard buffer solution the entire experimental period, and submitted only to the centrifugations in order to ensure that all cells undergo equal mechanical damage [8], [14].

### Cell viability

Cell viability was assessed by relative fluorescence of 50 µM ethidium bromide (Sigma-Aldrich) using a Hitachi F4500 spectrofluorometer at excitation and emission wavelengths of 365 and 580 nm, respectively [33]. Cells were treated with 0.005% digitonin at the end of each experiment to promote 100% cell permeabilization. The auto-fluorescence of ethidium bromide was subtracted from total fluorescence in the presence of cells, ethidium bromide or digitonin. Data are expressed as the percentage of total cells [8], [14].

### Isolation of rat heart mitochondria

Heart mitochondria were isolated from adult male Wistar rats as described by Kowaltowski *et al*. [34]. Mitochondria were kept over ice until the experiments were initiated. To ensure mitoK_ATP_ activity and its pharmacological regulation, all experiments using isolated mitochondria were conducted within 1 h of isolation [14], [35].

### Oxygen uptake measurements

Oxygen consumption was measured in a 1.4 mL temperature-controlled vessel equipped with a magnetic stirrer, using a Clark-type electrode (Yellow Spring Instruments Company). Mitochondria (0.5 mg/mL) were incubated in medium (37°C) containing 125 mM sucrose, 65 mM KCl, 10 mM HEPES, pH 7.2, 2.5 mM KH_2_PO_4_ and 0.4 mM EGTA. Respiratory chain activity was maintained using a mixture of NAD-linked substrates (malate, glutamate, α-ketoglutarate and pyruvate, 1.25 mM each) or 2.5 mM succinate plus 2 µM rotenone.

### Mitochondrial Ca^2+^ transport

Variations in medium free Ca^2+^ concentrations were examined by measuring changes in the absorbance spectrum of arsenazo III (40 µM) using an SLM Aminco DW2000 spectrophotometer (SLM Instruments, Inc., Urbana, USA) set at the 675–685 nm wavelength pair [36].

### Western Blots

Protein fractions from HL-1 myocytes cells were subjected to 12% SDS-PAGE and transferred to a nitrocellulose membrane. Blots were blocked with 5% bovine serum albumin (BSA) in TBS-T (0.05% Tween 20 in 50 mM Tris–HCl (pH 7.4), 150 mM NaCl) and incubated overnight with a rabbit polyclonal antibody specific for mouse AKT (Calbiochem) at 0.2 µg/mL or mouse phospho-Akt (Cell Signaling) at 0.1 µg/mL in 0.1% BSA TBS-T. After primary antibody incubation, the blots were washed and incubated with peroxidase-conjugated secondary antibody (10 ng/mL, Calbiochem). The signal was developed with the SuperSignal West Pico Chemiluminescent Substrate kit (Pierce Biotechnology, Rockford, IL). Image densitometry was performed using Image J and Image Quant softwares.

### Mitochondrial swelling

Mitochondrial swelling was estimated from the decrease in absorbance of the mitochondrial suspension measured at 520 nm using a temperature-controlled SLM Aminco DW-2000 spectrophotometer equipped with continuous stirring at 37°C. Swelling of freshly isolated mitochondria was measured soon after their addition to K^+^-rich hyposmotic buffers. This procedure allows for a magnified measurement of K^+^ uptake due to prior K^+^ depletion during the mitochondrial isolation procedure [34]. Where indicated, experiments were conducted in media in which KCl was substituted by LiCl, and the solution pH was corrected using NaOH, as a control for K^+^-specificity. Mitochondrial light scattering changes 40 sec after the addition in the experimental buffer were used to generate the data shown in the figure.

### Data analysis

Experiments depict typical traces or averages±standard errors of the mean from at least 3 identical repetitions using different preparations. Data were compared by one-way ANOVA followed by Tukey's post-hoc test performed by OriginPro 7.5 SRO (OriginLab Corporation, Northampton, MA, USA). When one parameter was compared between two groups, Student's t-test was used.

## Results

Perfused rat hearts were pre-treated with different concentrations of PD153035 and submitted to 40 min ischemia followed by reperfusion. **Figures 1A–D** show representative left ventricular pressure measurements in these perfused hearts. Upon global ischemia, the contractile function of the isolated rat hearts ceased within a few cycles (**Panel A**). Following reperfusion, spontaneous beating is resumed, but with increases in diastolic pressures and decreased systolic performance, as indicated by the marked reduction in the developed pressure. On the other hand, hearts pre-treated with increasing PD153035 concentrations (10 pM, **Panel B**; 1 nM, **Panel C** or 100 nM, **Panel D**) presented significantly less increases in the diastolic pressure and reductions in the systolic performance. **Figures 1E–F** shows average left ventricular developed pressures (**Panel E**) and diastolic pressures (**Panel F**) in hearts submitted to ischemia/reperfusion in the presence of 10 pM (▴), 1 nM (○) or 100 nM PD153035 (♦). Compared to controls (□), PD153035 treatment strikingly improved cardiac function, with a maximal effect observed at 1 nM.

**Figure 1:** PD153035 improves cardiac function after ischemia/reperfusion. **Panels A–D**: Perfused rat hearts were submitted to left ventricular pressure measurements after 15 min stabilizing perfusion, as described in the Methods section. PD153035 was present at 10 pM, 1 nM or 100 nM (**Panels B**, **C** and **D**, respectively) during the full experimental period. **Panel A** shows hearts in the absence of PD153035. After 10 min, the hearts were submitted to 40 min ischemia by interruption of coronary flow, followed by 35 min reperfusion. Data are representative traces of 3 similar repetitions. LVP: Left ventricular pressure. **Panels E–F**: Averages±SEM of 3 experiments conducted under the conditions of Panels A–D. DLVP: developed left ventricular pressure; DP: diastolic pressure. Values for 10 pM, 1 nM and 100 nM PD153035 concentrations were significantly different from controls at 85 min (*p*<0.05).

The cardioprotective effects of PD153035 were confirmed using a cultured cell model involving murine cardiac HL-1 cells, which allows for direct measurements of cell death [14], [31]. In these cells, metabolic inhibition promoted by treatment with cyanide and 2-deoxyglucose, followed by return to control conditions, mimics cardiac ischemia/reperfusion (**Figure 2A**, ⋄). Indeed, cell death occurs predominantly after the return of metabolic activity (the simulated reperfusion period which begins where indicated by the second arrow) [14]. The presence of 10 nM PD153035 in the preincubation media completely abrogated cell death promoted by cyanide/aglycemia in cardiac HL-1 cells (▴), while an equal quantity of the compound's solvent, DMSO (0.05%), had no protective effect (▪).

**Figure 2:** PD153035 protects against cardiac cell damage promoted by cyanide/aglycemia. **Panel A**: Cardiac HL-1 cells were preincubated in standard media (see Materials and Methods) containing 10 nM PD153035 (▴), the equivalent concentration of PD153035 solvent DMSO (0.05%; ▪) or no further additions (○, ⋄). Where indicated, all cells except controls (○) were treated with 10 mM K-cyanide (CN) and 2 mM 2-deoxyglucose (2-DG). All cells were submitted to equal centrifugations and media changes where indicated by the arrows. **Panel B** represents average cellular viability at 140 min. HL-1 cells were treated as described in Panel A. Where indicated, cells were preincubated in the presence of 60 µM 5-hydroxydecanoate (5HD) and/or 10 nM PD153035 (PD). Data represent average cell viability (see Materials and Methods) of 5 experiments±SEM. Data in Panels A and B represent separate experimental groups in which baseline measurements are not significantly distinct. *p<0.05 relative to “control” and “CN+2-DG+PD153035” at the respective time point. ^#^ *p*<0.05 relative to “CN+2-DG” at the respective time point.

Under these conditions, HL-1 cell death is dependent on the induction of the permeability transition, a Ca^2+^-induced non-selective inner mitochondrial membrane permeabilization [5], [6], [8]. In order to verify if inhibition of mitochondrial permeability transition was involved in the cardioprotective effects of PD153035, we tested if this compound could inhibit this process in isolated rat heart mitochondria (**Figure 3**). Mitochondria are able to take up large quantities of Ca^2+^, followed by release of this ion due to non-selective permeabilization (*line a*). The presence of the permeability transition inhibitor cyclosporin A prevents Ca^2+^ release without affecting uptake (*line b*). On the other hand, PD153035 did not inhibit either Ca^2+^ uptake or release at nanomolar (*lines c–f*) or micromolar concentrations (up to 40 µM, results not shown).

**Figure 3:** PD153035 does not decrease mitochondrial Ca^2+^ uptake, nor prevent permeability transition. Isolated rat heart mitochondria (RHM; 0.5 mg/mL) were incubated in 125 mM sucrose, 65 mM KCl, 10 mM HEPES, 2.5 mM KH_2_PO_4_, 40 µM arsenazo III, 1.25 mM malate, 1.25 mM glutamate, 1.25 mM pyruvate and 1.25 mM α-ketoglutarate, pH 7.2 (KOH). Ca^2+^ was added where indicated in four consecutive boluses of 10 µM, totaling 40 µM. *Line a* represents a control experiment with no further additions. *Line b* represents an experiment conducted in the presence of 1 µM cyclosporin A. *Lines c–f* represent experiments conducted in the presence of 1 nM, 10 nM, 30 nM and 100 nM PD153035, sequentially. Data are representative traces of 3 similar repetitions.

Since mitochondria are intimately involved in ischemic cardioprotection [1]–[3], [7], [8], [12] we also investigated if PD153035 affected respiration and oxidative phosphorylation in these organelles. We found that nanomolar PD153035 concentrations did not affect mitochondrial respiratory rates in the presence (state 3) or absence (state 4) of oxidative phosphorylation using NADH-linked substrates (**Table 1**) or succinate plus rotenone (results not shown). PD153035 also did not affect ATP synthesis, as determined by the lack of change in respiratory control and ADP/O ratios.

**Table 1:** PD153035 does not change mitochondrial respiratory parameters.

	Control	PD153035
State 3 respiratory rate (nmol O_2_×mg protein^−1^×min^−1^)	113.4±8.9	109.9±7.3
State 4 respiratory rate (nmol O_2_×mg protein^−1^×min^−1^)	16.21±1.59	16.93±1.27
Respiratory control ratio (state 3/state 4)	7.25±0.46	6.58±0.23
ADP/O ratio	2.06±0.14	2.14±0.12

Rat heart mitochondria were incubated in 125 mM sucrose, 65 mM KCl, 10 mM HEPES, 2.5 mM KH_2_PO_4_, 0.4 mM EGTA, 1.25 mM malate, 1.25 mM glutamate, 1.25 mM pyruvate and 1.25 mM α-ketoglutarate, pH 7.2 (KOH), in the presence of 10 nM PD153035 or the equivalent concentration of PD153035 solvent DMSO (0.1%) (Control), as indicated. ADP (250 µM) and 1 µg/mL oligomycin were added to achieve state 3 and 4 respiratory rates, respectively. Respiration was measured using a Clark-type electrode, and respiratory parameters were calculated as described in Materials and Methods. None of the values obtained in the presence of PD153035 are significantly different from controls (four independent preparations, experiments performed in triplicate).

An important phenomenon involved in cardioprotection in both ischemic/reperfused hearts and cyanide-treated/aglycemic cardiomyocytes is the activation of mitochondrial ATP-sensitive K^+^ channels (mitoK_ATP_) [2], [37]. Indeed, we found that cytoprotection promoted by PD153035 could be completely abrogated by mitoK_ATP_ inhibitor 5-hydroxydecanoate (5HD), which had no effect on the survival of control cells or cyanide/aglycemic cells not treated with PD153035 (**Figure 2B**). This finding leads to the hypothesis that PD153035 could activate mitoK_ATP_. To further study the activation of mitoK_ATP_ under our experimental conditions, we tested if this channel could be activated via intracellular signaling involving the PI3K-AKT cascade [20], [21] or directly via activation of mitoK_ATP_. We found that AKT levels were similar under all conditions, while pAKT (the active form) decreased to undetectable levels with cyanide/aglycemia. No evidence for AKT activation by PD153035 treatment was obtained either in control or cyanide-treated/aglycemic cardiomyocytes (**Figure 4**).

**Figure 4:** PD153035 does not alter AKT phosphorylation. Cardiac HL-1 cells were preincubated in standard media (see Materials and Methods) containing 10 nM PD153035 or the equivalent concentration of PD153035 solvent DMSO during 20 min. 10 mM K-cyanide (CN) and 2 mM 2-deoxyglucose (2-DG) were then added under the conditions of Figure 2, where indicated. After 60 min, suspension proteins were extracted and AKT and pAKT levels were estimated by immunoblotting. *p<0.01 relative to the conditions in the absence of “CN+2-DG”.

In order to test if PD153035 could directly activate mitoK_ATP_, we added this compound directly to isolated mitochondria and followed organellar swelling due to K^+^ uptake, which is accompanied by the uptake of phosphate and water [37]. Under these conditions, mitoK_ATP_ agonist diazoxide (DZX) reversed ATP-inhibited mitochondrial swelling in K^+^ media, in a manner inhibited by 5HD (results not shown; [16]). Interestingly, PD153035 partially reversed the inhibitory effect of ATP on mitochondrial swelling (see **Figure 5A** for typical traces and **5B** for averages). More strikingly, PD153035 increased swelling under control conditions in K^+^, but not Li^+^, media (**Figure 5B**). This indicates that PD153035 increases overall mitochondrial ATP-sensitive K^+^ transport activity. The activation was prevented by mitoK_ATP_ inhibitor 5HD (**Figure 5B**), which does not affect swelling under control conditions [16]. The equivalent concentration of PD153035 solvent DMSO (0.1%) had no significant effect on mitochondrial swelling (not shown).

**Figure 5:** PD153035 increases mitochondrial ATP-sensitive K^+^ transport. Isolated rat heart mitochondria (RHM; 0.5 mg/mL) were suspended in 100 mM KCl, 5 mM HEPES, 2 mM P_i_, 1 mM MgCl_2_, 0.1 mM EGTA, 1 µg/mL oligomycin and 10 mM succinate, pH 7.4 (KOH), and light scattering changes were recorded over the first 40 seconds. Where indicated, 200 µM ATP, 10 nM PD153035, 20 µM DZX and/or 60 µM 5-HD were present. Control experiments were conducted in the presence of the equivalent concentration of PD153035 solvent DMSO (0.1%). **Panel A** depicts representative traces, while **Panel B** shows average±SEM swelling relative to control of 8 experimental repetitions. The hatched column represents an experiment in which KCl was substituted by LiCl. *p<0.01 versus control; ^#^ *p*<0.01 versus PD. The effect of PD153035 in Li^+^ media was compared to swelling in Li^+^ media in the absence of this drug. Incubations in Li^+^ media resulted in 88.6±4.0% of the swelling observed in K^+^ media.

## Discussion

We demonstrate here that the 4-anilinoquinazoline derivative PD153035 is a potent cardioprotective agent capable of preventing reperfusion injury when used in the nanomolar concentration range (**Figure 1**). Furthermore, nanomolar concentrations of PD153035 completely prevented cardiac HL-1 cell death promoted by metabolic inhibition followed by a return of oxidative metabolism (**Figure 2**), a situation in which cellular damage occurs through mechanisms similar to those found in ischemia/reperfusion [8], [14].

Cytoprotection by PD153035 was completely reversed by 5HD (**Figure 2B**), an antagonist of mitoK_ATP_ channels. These channels are well known mediators of ischemic cardioprotection promoted by preconditioning or other known cardioprotective drugs [2], [12]. In fact, when tested in isolated mitochondria, PD153035 activated K^+^ uptake in an ATP-sensitive, 5HD-inhibited manner (**Figure 5**). No effects of PD153035 were observed in media in which K^+^ ions were substituted by Li^+^. Together, these data suggest that PD153035 directly activates a K^+^-selective, ATP-sensitive transport typical of mitoK_ATP_. On the other hand, we found no significant effect of PD153035 on oxidative phosphorylation (**Table 1**), mitochondrial Ca^2+^ uptake and retention (**Figure 3**) or AKT phosphorylation (**Figure 4**). These results indicate that the direct activation of mitoK_ATP_ by PD153035 can explain cardioprotection by this compound, although cardioprotection may also involve increases of this channel's activity by AKT-independent intracellular signaling events initiated by this compound's inhibitory effect on EGF receptor tyrosine kinase. Interestingly, although EGF tyrosine kinase 2 is a survival factor for human cardiomyocytes [22], not all inhibitors of this kinase present overt cardiotoxicity [38].

MitoK_ATP_ are highly K^+^-selective channels, which promote uptake of this ion down the mitochondrial electrochemical gradient. Transport through these channels is inhibited physiologically by ATP and ADP, and activated by GTP, GDP and UDP [39], [40]. Many pharmacological agonists and antagonists for these channels have been studied [41]. In particular, diazoxide (DZX) is widely used as a mitoK_ATP_ agonist due to its selectivity toward mitochondrial, and not plasma membrane, ATP-sensitive K^+^ channels [37]. DZX is capable of overcoming the inhibitory effect of ATP or ADP on mitoK_ATP_. Similarly, 5-hydroxydecanoate (5HD) is a mitoK_ATP_ antagonist with no measurable effect on sarcolemal K^+^ transport [16]. 5HD prevents the agonistic effect of DZX and other physiological and pharmacological mitoK_ATP_ activators.

The mechanisms through which mitoK_ATP_ promotes ischemic cardioprotection are complex and still remain to be completely understood. MitoK_ATP_ activity is capable of preventing loss of cellular high energy phosphates, resulting in a more favorable energetic state [42], [43]. The channel activation also prevents excessive Ca^2+^ uptake in mitochondria exclusively during ischemia, when this uptake is supported by ATP hydrolysis by the ATPsynthase [42], [44], [45]. This inhibition of Ca^2+^ uptake, in association with a decrease in mitochondrial oxidative stress also promoted by mitoK_ATP_ activity, results in prevention of mitochondrial permeability transition and ensuing loss of organellar functionality [2], [8].

Although DZX is a useful tool for *in vitro* mitoK_ATP_ studies, this drug has limited applicability for *in vivo* myocardial protection, since its effect on pancreatic islet K^+^ channel transport results in decreases in insulin secretion [46]. Furthermore, a desirable mitoK_ATP_ agonist should be active at very low concentrations, preferably less than the micromolar range necessary for DZX to activate mitoK_ATP_. Interestingly, Prada et al [47] recently showed that treatment with PD153035 reduces levels of inflammatory markers and improves glucose tolerance, insulin sensitivity and signaling in high-fat diet-fed mice.

The direct activation of mitoK_ATP_ by PD153035 in isolated mitochondria was a surprising finding of the present study, since this compound bears no strong structural resemblance with any known mitoK_ATP_ agonist [12]. On the other hand, PD153035 is a kinase inhibitor due to its ability to prevent ATP binding to these enzymes [28]. Since mitoK_ATP_ is also inhibited by ATP and ADP, it is tempting to speculate that PD153035 activates the channel by interfering with binding of these nucleotides to the protein. Interestingly, PD153035 is, to our knowledge, the only compound capable of activating mitochondrial K^+^ uptake in the absence of added ATP or ADP, possibly due to displacement of endogenous adenine nucleotides. This unique characteristic may render the drug more effective as an agonist.

4-anilinoquinazoline derivatives are currently believed to be viable clinical tools for control of proliferative diseases such as cancer and psoriasis, and act by inhibiting the EGF receptor family of tyrosine kinases [48]–[51]. Indeed, ^11^C-PD153035 can be used as an EGF receptor tracer in whole-body examinations for cancerous tissue, and has already been successfully tested in humans [52]. Quinazoline derivatives also act as antagonists of α-adrenergic receptors and may be used as anti-hypertensives [53]. Our results uncover another potential application for PD153035, as a powerful protective agent in ischemic heart disease. Furthermore, our results demonstrate that this compound is capable of substantially activating mitochondrial ATP-sensitive K^+^ uptake.
